The article "ECG Heartbeat Classification Based on an Improved ResNet-18 Model" was published in 2021. Journal: Comput Math Methods Med.

# ECG Heartbeat Classification Based on an Improved ResNet-18 Model

**DOI:** 10.1155/2021/6649970

**Published:** 2021-04-30

**Authors:** Enbiao Jing, Haiyang Zhang, ZhiGang Li, Yazhi Liu, Zhanlin Ji, Ivan Ganchev

**Affiliations:** ^1^College of Artificial Intelligence, North China University of Science and Technology, China; ^2^Department of Computer Science, University of Sheffield, UK; ^3^Telecommunications Research Centre (TRC), University of Limerick, Limerick, Ireland; ^4^Department of Computer Systems, University of Plovdiv “Paisii Hilendarski”, Plovdiv, Bulgaria; ^5^Institute of Mathematics and Informatics-Bulgarian Academy of Sciences, Sofia, Bulgaria

## Abstract

Based on a convolutional neural network (CNN) approach, this article proposes an improved ResNet-18 model for heartbeat classification of electrocardiogram (ECG) signals through appropriate model training and parameter adjustment. Due to the unique residual structure of the model, the utilized CNN layered structure can be deepened in order to achieve better classification performance. The results of applying the proposed model to the MIT-BIH arrhythmia database demonstrate that the model achieves higher accuracy (96.50%) compared to other state-of-the-art classification models, while specifically for the ventricular ectopic heartbeat class, its sensitivity is 93.83% and the precision is 97.44%.

## 1. Introduction

With the acceleration of the economy, the incidence and mortality of cardiovascular diseases (CVDs) have continued to increase in recent years, and the trend is becoming more and more obvious, especially for young people. CVDs are the number one cause of death worldwide. Arrhythmia is very common and can lead to cardiac arrest or even death [1]. According to World Health Organization (WHO), most patients with acute CVDs have a clinical manifestation of loss of consciousness after the onset of symptoms and, if not treated, they may die within 24 hours [2]. Therefore, the accurate and timely detection of patients' abnormal heartbeats in electrocardiograms (ECGs) has become an important problem for addressing in the medical field.

Some arrhythmia types are very rare [3], so patients must be monitored for a long time to identify the type of arrhythmia. ECG has been used as the main method for diagnosing CVDs [4], which is of great significance in the detection of arrhythmia. The ECG signal consists of three waves—P wave, QRS wave, and T wave [5], as shown on Figure 1.

Arrhythmia types can generally be divided into two categories. The first one includes life-threatening arrhythmia types, such as ventricular fibrillation and tachycardia. These arrhythmias require immediate treatment and have been well studied [6]. The second category is not immediately life-threatening but still need to be investigated and treated accordingly. In this category, arrhythmia is caused by a single irregular heartbeat, and the interval and amplitude defined by the ECG features contain most of the clinically useful information. This means that the shape of the ECG signal and other morphological characteristics determine the type of arrhythmia [7].

In clinical practice, the changes of ECG parameters are identified by doctors based on visual evaluation and manual interpretation methods in order to detect CVDs. Due to the nonstationary and nonlinear nature of ECG signals, however, CVD indicators may appear randomly on the time scale [8]. This and other factors make the classification of arrhythmic heartbeats in ECG signals a very challenging and time-consuming task, and so, it is almost unrealistic to perform it manually. Therefore, automatic classification approaches that analyze the records and classify the types of heartbeats have become very important.

In the past few decades, in the area of artificial intelligence (AI), researchers have developed different machine learning (ML) and deep learning (DL) techniques to classify arrhythmias. Among the latter, artificial neural networks are quite popular for classification, pattern recognition, feature extraction, and so on. There are different types of neural networks. Convolutional neural networks (CNNs) have been developed in recent years to classify massive data. In this article, a CNN approach is applied for the classification of ECG heartbeats for the purposes of identifying arrhythmia cases.

The main contributions of this article are the following:

1. Wavelet transform is used for denoising the ECG signals, due to its high resolution of time and frequency, allowing it to successfully recognize the abstract and hidden features of ECG signals [8]
2. An improved version of the ResNet-18 model [9] is elaborated and proposed for ECG heartbeat classification, with an ability to extract features in depth
3. A performance comparison of the proposed model with state-of-the-art models is presented, based on experiments conducted with the Massachusetts Institute of Technology-Boston's Beth Israel Hospital (MIT-BIH) arrhythmia database, showing that the proposed model achieves the highest classification accuracy among the models compared

The rest of this article is structured as follows.  Section 2 introduces the related work done in the ML/DL area for ECG monitoring.  Section 3 presents background information about ECG signals, CNNs, and residual networks (ResNet).  Section 4 describes the proposed model along with its training algorithm and parameters.  Section 5 presents and discusses the performance comparison results obtained from the conducted experiments. Finally, Section 6 concludes the article.

## 2. Related Work

In recent years, AI has been applied to the field of ECG signal analysis. Various ML, and especially DL, techniques have shown good success in finding abnormal ECG waveforms and events, thereby improving the detection accuracy of a variety of heart-related diseases. In terms of data processing, one possible approach is to treat the ECG signal as one-dimensional (1D) data and process it according to the standard method applied to an ordinary text [10]. Tamás et al. [11] used a Hermitian matrix and wavelets to carry out adaptive orthogonal transform on patient features. By using ensemble learning technology to train the processed data, this method shows potential in arrhythmia detection. Chazal et al. [12] divided the MIT-BIH data set into the independent training set and test set, which makes the evaluation results more objective and in line with reality. Saini et al. [13] divided the pulsation of an ECG signal into four categories and proposed a support vector machine (SVM) model, based on empirical mode decomposition and multicategory directed acyclic graph. Thomas et al. [14] performed a dual-tree complex wavelet transform on an ECG data and realized an automatic extraction of features.

The recently emerged DL models are powerful, even though computationally expensive, analytical models that can greatly reduce the use of artificial features [8]. DL models are based on the use of deep neural networks (DNNs), which are subdivided into convolutional neural networks (CNNs), recursive neural networks (RNNs), and long-term short-term memory (LSTM). Among these, CNNs are widely used in many fields. One of the most important features of a CNN is that its complex structure provides a certain degree of translation, scaling, and rotation invariance, because the local receptive field allows neurons or processing units to access underlying features, such as directional edges or corners. Therefore, the CNN-based approach demonstrates very good performance in classification of ECG signals, especially to solve prediction problems in ECG arrhythmia classification, due to its strong robustness and fault tolerance to noise [8]. Xu et al. [15] used a DNN to classify ECG signals end-to-end, demonstrating by this the possibility for complete intelligence of ECG analysis [8]. Yande et al. [16] proposed a two-layer CNN to distinguish the R-R interval (the interval between two successive R waves of the QRS complex wave, c.f. Figure 1). Hannun et al. developed an algorithm based on a 34-layer CNN [17] to detect various arrhythmias by using single-lead ECG data generated by sensing/monitoring equipment. The diagnostic performance of this algorithm can exceed that of an ordinary cardiologist in detecting distinct arrhythmias, which could be attributed to the feature learning capability of DNN, realizing the function of feature extraction and classification [8]. Jiang and Seong Kong specially designed a block-based neural network [18]. Sellami and Hwang [19] proposed a robust deep CNN with a batch weighted loss.

Although results from the aforementioned works are significant, deeper features cannot be extracted because of the limitation on the number of neural network's layers. Naturally, the learning ability of a neural network increases with the number of its layers. However, deepening the network may produce gradient dissipation restricting its performance [8] and preventing it to converge. To cope with this, the ResNet structure [9] seems to be a good choice employed by researchers working in this field. For instance, Zhou et al. [20] proposed an attention mechanism based on ResNet for ECG data processing, using two commonly used databases—the MIT-BIH database and the Physikalisch-Technische Bundesanstalt diagnostic ECG database (PTB), which stands out in both databases. Park et al. [21] proposed a SE-ResNet, a residual network with a squeeze-and-excitation block, which outperforms the ResNet baseline model. Han et al. [22] used a multilead residual neural network (ML-ResNet) with three residual blocks and feature fusion to detect and locate myocardial infarction using 12 leads ECG records.

## 3. Background

### 3.1. ECG Signals

#### 3.1.1. MIT-BIH Arrhythmia Database

One of the most commonly used databases in the world, used as a source of clinical ECG signals, is the MIT-BIH database, which is divided into several subsets. One of these is the MIT-BIH arrhythmia database [23], which is the more widely used in this field [8]. It consists of 48 half-hour two-channel ambulatory ECG signal recordings of 47 subjects, digitized at a frequency of 360 samples per second per channel with 11-bit resolution, over a 10 mV range. 25 male subjects, aged 32 to 89, and 22 female subjects, aged 23 to 89, participated for the creation of the database. 60% of the subjects were inpatients. Each record was annotated independently by two cardiologists to obtain approximately 110,000 computer-readable reference annotations for each beat, included in the database [23].

In the MIT-BIH database, there are 15 heartbeat types mapped to the 5 main classes of the AAMI standard [24], as shown in Table 1.

#### 3.1.2. ECG Signal Denoising

ECG signals are usually interfered by various noises such as baseline drift, electromyographic noise, electrode contact noise, powerline interference, motion artifacts, and instrument noise [25]. These noises can lead to incorrect diagnostic or wrong classification. For denoising an original ECG signal, wavelet transform could be used, as a suitable tool for all frequency ranges, resulting in an improvement of accuracy both in the time and frequency domains [8], as follows [26]:

(1) $$\begin{array}{c} WT\left(\text{a},\tau \right)=\frac{1}{\sqrt{a}}\int_{-\infty }^{\infty }f\left(\text{t}\right)*\Psi \left(\frac{t-\tau }{a}\right)dt, \end{array}$$

where *τ* represents the translation variable and a represents the scale variable. After translation and scaling, the wavelet transform can not only know the frequency components of the signal but also analyze the specific locations of different frequencies on the time scale for later calculations. Compared to Fourier transform, for instance, wavelet transform provides a variable time-frequency window, allowing dynamical change of its scale [8].

The commonly used nonlinear threshold method was selected to process ECG data in the experiments, conducted by us. The whole process of denoising ECG signals is depicted on Figure 2.

There are different wavelet bases, each with its own specific characteristics making it suitable to a specific application [27], e.g., Morlet, Mexican hat, Meyer, Daubechies, Symlets, Coiflets, Haar, and Biorthogonal wavelets. Choosing the most suitable wavelet base with an appropriate number of decomposition levels is vital for the proper signal denoising [8]. In the conducted experiments, the Daubechies wavelet base was utilized due to its energy spectrum symmetry (mainly around low frequencies) that is found more suitable for R peak identification, which is important for detection of tachycardia [8]—one of the life-threatening arrhythmia types. Within the Daubechies base, the db8 wavelet was selected as this performs best for ECG signals, compared to other wavelets [28]. In addition, a soft threshold was utilized as it shrinks the large magnitude wavelet coefficients above the threshold resulting in more smoothened and continuous output [29]. Due to the high fluctuation of the ECG signals, 9 levels were used for the wavelet decomposition, whereas the wavelet coefficients of each level were retained for the wavelet reconstruction.

Figure 3 shows the noise reduction effect on a random piece of patient data (the record with serial number 100) of the MIT-BIH arrhythmia database. In particular, it shows the removal of high-frequency noise, such as muscle artifacts, powerline interference, and electromyographic noise, which drastically distorts both temporal and spectral characteristics of the ECG signal [8]. The removal of muscle artifacts (without distorting the clinical features), for instance, is a very important task for recognizing various ECG arrhythmias [30]. Similarly, the removal of powerline interference will positively impact the diagnosis of atrial arrhythmias due to minimizing the P wave distortions [31]. Although the high-frequency noise is removed, the basic features of the ECG waveform are retained, which is convenient for the model training.

For single sample extraction, we used direct signal slicing, whereby each slice is 3 sec long. This value was chosen as a good compromise when compared to other values used in practice, as shorter slice duration may lead to incomplete waveform information interception, while longer slice duration may contain more waveforms, affecting the neural network's detection ability. For instance, as shown in [32] for a similar CNN-based arrhythmia detection method, the use of 2 sec and 5 sec slice durations results in accuracy of 92.50% and 94.90%, respectively, while with 3-sec slices our model achieves higher accuracy of 96.50%.

The following rules were adopted for slice labeling:

1. If all heartbeats in a slice are normal, the slice is considered normal as well
2. If both normal and abnormal heartbeats are present in a slice, the slice is considered abnormal
3. If multiple types of abnormal heartbeats are present in a slice, the most represented abnormal type defines the slice type
4. In the case of a tiebreak, i.e., having multiple types of abnormal heartbeats with the same number of representations in a slice, the first anomaly type appearing in the slice defines the slice type

It is worth mentioning that, in order to increase the number of samples, the method of slice overlapping was applied. This is justified because the advantages of the slicing method outweigh the disadvantages—the captured information is more complete, it does not depend on a specific QRS detection algorithm, and the entire process is simplified. The slices were made from the beginning of the record to ensure full utilization of the data set, which is of great significance for increasing the robustness of the model.

#### 3.1.3. ECG Signal Classification

The approach used for ECG signal classification is similar to the one applied for image classification, which seeks deep-seated features by increasing the number of DL layers. Therefore, our research was focused on finding a DL model suitable for ECG multiclassification by changing the ResNet hierarchy. This article presents the achieved result—an improved version of the ResNet-18 baseline model for CNNs. Due to the ResNet-18 characteristics, the CNN can extract more features by increasing the number of convolutional layers while achieving an improved accuracy. Single-lead ECGs from the MIT-BIH arrhythmia database were classified with the proposed model, which showed better performance compared to the existing state-of-the-art models in terms of both classification accuracy and computation time.  Figure 4 shows the process of heartbeat classification, utilized in our research.

In terms of input data, one of the methods used for ECG data classification is the interpatient method, which extracts and classifies features of different patients, whereby the patient data used in the test phase is not used to train the model. Another possibility is to use the intrapatient method, which directly allocates the data of the same patient in the training set and test set randomly [33]. It can be clearly seen that the classification of interpatient data is more realistic and meaningful. However, most of the current studies still rely on the intrapatient method. Although its classification accuracy is high, this is achieved by model training based on part of the ECG data of a patient, and then, model testing performed on the rest of data of the same patient. Therefore, this method is unreasonable and does not conform to the real situation.

The research presented in this article utilizes the interpatient data classification method. Accordingly, 44 out of the total 47 MIT-BIH records (patient data) were used in the conducted experiments. Out of these, 22 records were used as a test set. For cross-validation, the remaining records were split into two halves—one was used as a training set and the other as a validation set (Table 2).

### 3.2. CNNs and ResNets

Compared with traditional neural networks, CNNs have two characteristics, weight sharing and local connection, which greatly improve their ability to extract features and lead to improved efficiency and reduced number of training parameters. The main structure of a traditional CNN includes an input layer, a convolutional layer, a pooling layer, a fully connected layer, and an output layer, whereby the output of one layer serves as an input for the subsequent layer in the structure (Figure 5). Usually, the convolutional and pooling layers are alternately used in the structure.

The convolutional layer, the core of a CNN, contains multiple feature maps, whereby each feature map contains multiple neurons. When a CNN is used for image classification, for example, this layer scans the image through the convolution kernel and makes full use of the information of the adjacent areas in the image to extract image features. After using the activation function, the feature map of the image is obtained as follows [34]:

(2) $$\begin{array}{c} {\text{X}}_{j}^{l+1}=f\left(\underset{i\in M_{j}}{\sum }X_{i}^{l}*k_{ij}^{l+1}+b_{i}^{l+1}\right), \end{array}$$

where X_*j*_^*l*+1^ represents the *j*^th^ feature of the (*l* + 1)^th^ convolutional layer, *X*_*i*_^*l*^ represents the input characteristic, *f* represents the activation function (typically used is a rectifier linear unit, ReLU [35]), *M*_*j*_ represents a set of input feature maps, ∗ represents a convolution operation, *k* represents a convolution kernel, and *b* represents the offset term.

The role of the pooling layer, when used for image classification, is to imitate the human visual system to reduce the dimensionality of the data, and to represent the image with higher-level features as follows:

(3) $$\begin{array}{c} {\text{X}}_{j}^{l+1}=X_{j}^{l}⊗k_{j}^{l+1}+b_{j}^{l+1}, \end{array}$$

where ⊗ represents the pooling operation. The main pooling methods include maximum pooling, average pooling, and median pooling.

In the fully connected layer, the maximum likelihood function is used to calculate the probability of each sample, and the learned features are mapped to the target label. The label with the highest probability is used as the classification result to realize the CNN-based classification.

The deeper the CNN, the better its performance. However, with deepening the network, two major problems arise: (1) the gradient dissipates, which affects the network convergence, and (2) the accuracy tends to saturate. In order to solve the problems of gradient vanishing explosion and performance degradation caused by the depth increase, residual networks (ResNets) were proposed in [9], which are easier to optimize and can gain accuracy from considerably increased depth. The ResNet approach won the first place on the ILSVRC 2015 classification task [9].

Figure 6 depicts the ResNet building block with input parameter *x* and target output *H*(*x*). The block employs a shortcut connection allowing it to directly learn the residual *F*(*x*) = *H*(*x*) − *x* as to make the target output [*F*(*x*) + *x*], thus avoiding the problem of performance degradation and accuracy reduction due to having too many convolutional layers. Such shortcut connections can skip two or more layers and directly perform identity mapping.

It makes reference (*X*) for the input of each layer, learning to form a residual function, instead of learning some functions without reference (*X*). This residual function is easier to optimize and can greatly deepen the number of network layers. The ResNet building block in Figure 6 has two layers and uses the following residual mapping function [9]:

(4) $$\begin{array}{c} F=W_{2}\sigma \left(W_{1}x\right), \end{array}$$

where *σ* represents the activation function ReLU [35]. Then, through a shortcut connection and a second ReLU, one can get the output *y*:

(5) $$\begin{array}{c} y=F\left(x,\left\{W_{i}\right\}\right)+x. \end{array}$$

When a change of the input and output dimensions is needed (e.g., changing the number of channels), one can make a linear transformation *W*_*s*_ to *x* in the shortcut, as follows:

(6) $$\begin{array}{c} y=F\left(x,\left\{W_{i}\right\}\right)+W_{s}x. \end{array}$$

By using the ResNet building block, shown on Figure 6, residual networks of 18 and 34 layers (called ResNet-18 and ResNet-34, respectively) were proposed and evaluated in [9], where it was noted that ResNet-18 is comparably accurate as ResNet-34 but converges faster.

## 4. Proposed Model

The training of a neural network model requires a large number of data sets. When the amount of input data increases, the number of neurons in the model needs to be also increased as to improve the classification accuracy. A fully connected neural network increases in size with the increase of the input data dimension and the number of hidden layer neurons, which leads to the increase of network parameters, and as a result affects the training speed of the network model. As a solution to this problem, this article uses a CNN with characteristics of local connection and parameter sharing to reduce the number of model parameters and accelerate the training speed of the model. Lead ECG data are equivalent to one-dimensional time series. Therefore, the research method presented in this article enhances the CNN design with an improved ResNet-18 model for automatic classification in single-lead ECGs. The proposed model can extract multiple features of the ECG data from the same input, which results in efficient obtaining of the representation of the internal structure characteristics of the ECG data, thus improving the classification accuracy.

The elaborated improved ResNet-18 model was used to realize a high-precision identification and classification of the five AAMI heartbeat classes, based on the MIT-BIH arrhythmia database. Before preprocessing and training the CNN, the model must be compiled. Parameters are declared for calculation during training, such as the optimizer, the loss function, and the learning rate. The optimizer and the loss function are the key elements that enable the CNN to process data properly. The setting of the optimizer determines the learning rate of the neural network. The optimizer used in the elaborated model presented here is the stochastic gradient descent (SGD) [36], proven to perform better than many other optimizers. The loss function is an important criterion to measure the classification quality of the model. The proposed model uses the cross-entropy loss function [37]. The initial value of the learning rate is set to 0.1, and a step change is adopted in the follow-up, presenting a convenient way for the objective function to converge better.

The ECG data were sliced to obtain 1080 sampling points within a 3 sec window. The number of convolution kernels starts at 12 and then increases when passing through each convolutional layer. Since the improved ResNet-18 model is proposed here for identification of the five main AAMI classes (c.f. Table 1) in ECG signals, there are five output values.  Figure 7 shows the specific dimensions and values used in each layer.

For the input data, a one-dimension convolution kernel with a length of 32 is firstly used to extract the characteristics of the data. When the original ResNet-18 model is used for two-dimensional image classification, it tends to use a small convolution kernel with a size of 3 × 3. In general, the image resolution of the direct input network is relatively low. Even when the receptive field is at its minimum, the 3 × 3 region is likely to contain significant changes. The ECG signals are fundamentally different from the image data. For low-frequency, low-sampling signals such as ECGs, having only three sampling points at any given location leads to difficulties in forming a meaningful waveform change. In addition, these signals are highly susceptible to noise interference, which could have a significant negative impact on feature learning and, in severe cases, can even cause ineffective learning. Therefore, the use of large convolution kernel is proposed here for the effective alleviation of this problem.

Figure 8 shows the structure of the elaborated improved ResNet-18 model, which consists of four parts: a convolutional layer, a classic ResNet-18 layer, an improved ResNet-18 layer, and a fully connected layer. The first part, the convolutional layer, is used mainly to perform basic feature extraction on the input data in order to prepare these for the next deeper level. The second part uses the classic ResNet-18, which is known as one of the best models used for ECG multiclassification. In this part, the input data are convoluted twice, and the modified linear unit, ReLU, is added between the two convolutions. ReLU zeros the output of some neurons, which makes the network sparse and reduces the interdependence of parameters. It also alleviates the occurrence of overfitting problems. On the other hand, the data before convolution are inputted into a maximum pooling layer, which divides the sample into feature regions and uses the maximum value in a region as the region representative to reduce the amount of calculation and the number of parameters. Finally, two kinds of data with the same dimension after different processing are added to complete the creation of the block module. The purpose of this step is to inherit the optimization effect of the previous step and make the model continuing to converge.

In order to achieve better performance, we use an improved ResNet-18 in the third part. A batch norm is added before the classical ResNet-18 structure to accelerate the training of the neural network, increase the convergence speed, and maintain the stability of the algorithm. The elaborated model goes through this structure seven times, and then, the data are sent to the fourth part, which is a fully connected layer.

Finally, the output data features are mapped from the fully connected layer to a one-dimension vector, and the vector is regressed by a *softmax* function [38] (also called a normalized exponential function), which is suitable for a multiobjective classification. The goal is to transform the output feature vector of the fully connected layer into an exponential function and map an *n*-dimension real number vector into another *n*-dimension vector by an exponential function. Finally, all the results are added and normalized to present the multiclassification results in the form of probability. The *softmax* function used is defined as

(7) $$\begin{array}{c} y=\text{signalsFeature},\\ p_{i}=\text{softmax}\left({\mathrm{lg}}_{i}\right)=\frac{e^{{\mathrm{lg}}_{i}}}{\sum_{i=0}^{n^{-1}}e^{{\mathrm{lg}}_{i}}},\\ {ls}_{i}=\overset{n^{-1}}{\underset{i=0}{\sum }}y_{i}*\ln p_{i}, \end{array}$$

where signalsFeature is the label of the corresponding classification heartbeat type image; *y* is the unique thermal code, where the corresponding position of the actual heartbeat class label is 1, and the remaining positions are 0; *n* is the classification number of ECG tags; *p*_*i*_ is the probability that the heartbeat sample belongs to the *i*^th^ value; *ls*_*i*_ is the loss function of the corresponding flame state category; and lg_*i*_ is the *i*^th^ value of the output vector logits, which is used to represent the probability of this classification result. When the training samples are convoluted, regularized, activated, and pooled, the output data features are mapped into a one-dimension vector from the fully connected layer, and the vector is calculated by the *softmax* function. Finally, the results of the heartbeat classification are presented in the form of probability.

It is important that the *l*_2_ regularization [39] is added to all convolutional layers and to the fully connected layer in the proposed model, in order to speed up the convergence speed of the network and limit the generation of overfitting phenomenon. The loss function of weight regularization is defined as

(8) $$\begin{array}{c} \text{Loss}={\left(\theta -W^{T}\text{x}\right)}^{2}+\alpha {\left\|\text{W}\right\|}^{2}, \end{array}$$

where *α* is the coefficient of regular term, W is the network weight, *θ* is the prediction value of the heartbeat category, x is the feature of the heartbeat sample data, and *T* is the number of weighted items.

Dropout (set to 0.5) was added to the convolutional layer for reducing the number of parameters and training time.

In the conducted experiments, the improved ResNet-18 model was used to classify heartbeats in ECG images, available from the MIT-BIH arrhythmia database. Although it is difficult for the human eye to distinguish certain areas in ECG images due to the density of time series, with the help of the elaborated model, one can easily identify the tags in each marker image. Compared with other classification models (c.f. next section), the proposed model can classify complex mixed wave images in a shorter computational time. Overall, for complex images, both the model training and testing time are reduced. The model training is done according to Algorithm 1.

## 5. Experimental Results and Discussion

The experiments were carried out by means of the PyCharm development tool. The computer hardware configuration used included an Intel(R) Core i5 CPU, a NVIDIA GeForce GTX 1060 GPU, and an 8 GB RAM. The computer operating system was Windows 10, and the programming environment included Python 3.7 along with the open-source ML framework TensorFlow.

In the experiments, the network model, achieving the highest overall classification accuracy, was saved and used for the evaluation based on the test set. 100 such iterations were performed.  Table 3 shows the total number of MIT-BIH heartbeats included in the experiments along with the corresponding number of these used only as a test set, for each AAMI heartbeat class. Figures 9 and 10 illustrate the model loss and classification accuracy, respectively, as a function of the number of iterations. From these two figures, one can observe that after the 50^th^ iteration, the model gradually converges, reaching stable accuracy and minimum loss at the 100^th^ iteration.

The results shown in Table 4, obtained from the experiments conducted with the MIT-BIH data sets, confirm that the improved ResNet-18 model, proposed in this article, outperforms (in terms of overall accuracy) the state-of-the art models used for heartbeat classification.

Table 5 shows the confusion matrix of the improved ResNet-18 model, proposed in this article.

In the training process of the model, various indexes should be considered comprehensively, and various experimental results should be reasonably analyzed. For multiclassification problems, sensitivity (Se) and precision (P+) are usually used to measure the model performance. Sensitivity (a.k.a. probability of detection or recall) measures the proportion of the actual positives that are correctly identified by a classification model as such. In our case, sensitivity is the percentage of the actual disease cases that are correctly judged by the model, reflecting the ability of the model to discover such cases. The precision (a.k.a. positive predictive value) is the fraction of relevant instances among the retrieved instances. In our case, it gives the probability of accurate prediction of the model. For disease diagnosis, it is more important to increase as much as possible the sensitivity of the classification model than to increase its precision, because the proper discovery of a CVD is more important than a misdiagnosis.

As can be seen from Table 6, although the accuracy of the proposed model is very high (c.f. Table 4), its sensitivity for some of the heartbeat classes (i.e., S and F) is still low, or even zero for the Q class, which is due to the existing imbalance of the AAMI heartbeat class data contained in the MIT-BIH arrhythmia database (c.f. Table 5). This problem may have a severe effect on the model training process, thus likely invalidating the neural network learning. To solve this, the method of slice overlapping was applied in the process of intercepting a single sample. This is justified especially when the number of samples is small, so as to relatively increase it.

Table 7 compares (in terms of sensitivity and precision) the proposed model to the state-of-the-art models, when applied for classification of the AAMI heartbeat classes V and S, which contain most arrhythmias.

## 6. Conclusions

In this article, an improved ResNet-18 model has been proposed for ECG heartbeat classification. Slicing technology has been used to label the data, which simplified its preprocessing. The obtained experimental results demonstrated that the improved ResNet-18 model can effectively be used to identify arrhythmia classes. Moreover, the results confirmed that the proposed model is superior to the state-of-the-art models considered, in terms of classification accuracy, by achieving the highest rate of 96.50%. Therefore, the model has great clinical application prospects and is worthy of further study and elaboration.

In order to reduce the impact of the heartbeat class imbalance on the performance of the model, one way is to increase the weight of a small class of losses by modifying the loss function, and to use the weighted loss, obtained through batch processing. Another idea could be to apply data enhancement, which increases the amount of data by cutting and splicing the ECG data to get a better training effect. Last but not least, some features for small categories could be introduced, so that the neural network can better identify small categories of abnormalities.

## Figures and Tables

**Figure 1:** Single heartbeat waveform.

**Figure 2:** ECG signal denoising process.

**Figure 3:** ECG signal comparison before denoising (red color) and after denoising (black color).

**Figure 4:** Heartbeat classification based on the proposed model.

**Figure 5:** The overall structure of a convolutional neural network (CNN).

**Figure 6:** The ResNet building block (adapted from [34]).

**Figure 7:** Parameters of each layer of the improved ResNet-18 model.

**Figure 8:** The structure of improved ResNet-18 model.

**Figure 9:** The improved ResNet-18 model's loss as a function of the number of iterations.

**Figure 10:** The improved ResNet-18 model's accuracy as a function of the number of iterations.

**Algorithm 1:** The training algorithm of the improved ResNet-18 model.

**Table 1:** Mapping of the MIT-BIH heartbeat types to the AAMI heartbeat classes.

AAMI heartbeat classes	MIT-BIH heartbeat types
Normal (N)	Normal beat Left bundle branch block beat Right bundle branch block beat Atrial escape beat Nodal (junctional) escape beat

Ventricular ectopic (V)	Premature ventricular contraction Ventricular escape beat

Supraventricular ectopic (S)	Atrial premature contraction Aberrated atrial premature beat Nodal (junctional) premature beat Supraventricular premature beat

Fusion (F)	Fusion of nonectopic and ventricular beat

Unknown (Q)	Paced beat Fusion of paced and normal beat Unclassifiable beat

**Table 2:** The training set, validation set, and test set used in the experiments.

Data sets	Serial numbers of MIT-BIH patient records
Training set	124, 201, 203, 205, 207, 208, 209, 215, 220, 223, 230
Validation set	101, 106, 108, 109, 112, 114, 115, 116, 118, 119, 122
Test set	100, 103, 105, 111, 113, 117, 121, 123, 200, 202, 210, 212, 213, 214, 219, 221, 222, 228, 231, 232, 233, 234

**Table 3:** The number of heartbeats, retrieved from the MIT-BIH database and used in the experiments, for each AAMI heartbeat class.

AAMI heartbeat class	Number of heartbeats retrieved from MIT-BIH	Number of MIT-BIH heartbeats used as a test set
N	73,564	36,727
V	24,122	12,219
S	3,880	1,835
F	586	300
Q	20	5
	102,172 (in total)	51,086 (in total)

**Table 4:** Performance comparison of different classification models, in terms of overall accuracy.

Model	Overall accuracy (%)
Ensemble learning [11]	94.20
BbNNs [18]	94.49 (calculated by us, based on the confusion matrix provided in [18])
End-to-end DNN [15]	94.70 (as the proportion of classes F and Q in the MIT-BIH data set is very small (less than 1%), these two classes have insignificant contribution to the overall performance and so they were not included in the calculation of the overall accuracy presented in [15])
1D-CNN [10]	95.13 (calculated by us, based on the confusion matrix provided in [10])
Improved ResNet-18 (the proposed model)	96.50

**Table 5:** The confusion matrix of the improved ResNet-18 model.

Actual AAMI heartbeat class	Predicted AAMI heartbeat class				
	N	V	S	F	Q
N	35617	680	419	9	2
V	139	11906	54	120	0
S	226	66	1539	4	0
F	33	34	1	232	0
Q	2	3	0	0	0

**Table 6:** Sensitivity (Se) and precision (P+) of the improved ResNet-18 model for each AAMI heartbeat class.

AAMI heartbeat class	Se (%)	P+ (%)
N	98.89	96.98
V	93.83	97.44
S	76.45	83.87
F	63.56	77.33
Q	0	0

**Table 7:** Sensitivity (Se) and precision (P+) of the improved ResNet-18 model, in comparison with state-of-the-art models, for AAMI heartbeat classes V and S.

Model (ensemble learning is omitted from this comparison as there are neither sensitivity nor precision data presented for it in [11])	AAMI heartbeat class V		AAMI heartbeat class S	
	Se (%)	P+ (%)	Se (%)	P+ (%)
BbNNs [18]	86.60	93.30	50.60	67.90
End-to-end DNN [15]	93.70	Not provided	77.30	Not provided
1D-CNN [10]	93.90	90.60	60.30	63.50
Improved ResNet-18 (the proposed model)	93.83	97.44	76.45	83.87

## Data Availability

The public data set, MIT-BIH Arrhythmia Database, is used and it can be accessed from https://www.physionet.org/.
